The article "Cord Blood Stem Cells Inhibit Epidermal Growth Factor Receptor Translocation to Mitochondria in Glioblastoma" was retracted in 2025. Reasons: duplicated images; overlap with earlier publications; unreliable results or conclusions; concerns about the images.

# Cord Blood Stem Cells Inhibit Epidermal Growth Factor Receptor Translocation to Mitochondria in Glioblastoma

**DOI:** 10.1371/journal.pone.0031884

**Published:** 2012-02-14

**Authors:** Venkata Ramesh Dasari, Kiran Kumar Velpula, Kiranmai Alapati, Meena Gujrati, Andrew J. Tsung

**Affiliations:** 1 Departments of Cancer Biology and Pharmacology, University of Illinois College of Medicine at Peoria, Peoria, Illinois, United States of America; 2 Department of Neurosurgery, University of Illinois College of Medicine at Peoria, Peoria, Illinois, United States of America; 3 Department of Pathology, University of Illinois College of Medicine at Peoria, Peoria, Illinois, United States of America; 4 Illinois Neurological Institute, University of Illinois College of Medicine at Peoria, Peoria, Illinois, United States of America; University of Udine, Italy

## Abstract

**Background:**

Overexpression of EGFR is one of the most frequently diagnosed genetic aberrations of glioblastoma multiforme (GBM). EGFR signaling is involved in diverse cellular functions and is dependent on the type of preferred receptor complexes. EGFR translocation to mitochondria has been reported recently in different cancer types. However, mechanistic aspects of EGFR translocation to mitochondria in GBM have not been evaluated to date.

**Methodology/Principle Findings:**

In the present study, we analyzed the expression of EGFR in GBM-patient derived specimens using immunohistochemistry, reverse-transcription based PCR and Western blotting techniques. In clinical samples, EGFR co-localizes with FAK in mitochondria. We evaluated this previous observation in standard glioma cell lines and *in vivo* mice xenografts. We further analyzed the effect of human umbilical cord blood stem cells (hUCBSC) on the inhibition of EGFR expression and EGFR signaling in glioma cells and xenografts. Treatment with hUCBSC inhibited the expression of EGFR and its co-localization with FAK in glioma cells. Also, hUCBSC inhibited the co-localization of activated forms of EGFR, FAK and c-Src in mitochondria of glioma cells and xenografts. In addition, hUCBSC also inhibited EGFR signaling proteins in glioma cells both *in vitro* and *in vivo*.

**Conclusions/Significance:**

We have shown that hUCBSC treatments inhibit phosphorylation of EGFR, FAK and c-Src forms. Our findings associate EGFR expression and its localization to mitochondria with specific biological functions in GBM cells and provide relevant preclinical information that can be used for the development of effective hUCBSC-based therapies.

## Introduction

Epidermal growth factor receptor (EGFR) expression in glioblastoma multiforme (GBM) has both diagnostic and prognostic significance [1]–[4]. EGFR signaling plays an important role in the formation and tumorigenicity of malignant gliomas, and EGFR overexpression can be found in 40 to 50 percent of patients with GBM [5]. Multiple histopathological and genetic studies, together with recent large-scale cancer gene sequencing efforts, have identified EGFR and its downstream signaling networks as commonly deregulated components in the primary GBM tumors [1], [6], [7]. Furthermore, substantial experimental evidence support a causal role for aberrant EGFR signaling in cancer pathogenesis and resistance to treatment [8]. GBM show very high resistance to treatment with radiation and chemotherapy and aberrant EGFR signaling contributes to this resistance. Thus, although initial attempts to target the EGFR have not been effective in GBM [9], EGFR remains an attractive target for therapeutic intervention in GBM.

Binding of the ligand epidermal growth factor (EGF) to EGFR triggers receptor dimerization and activates tyrosine kinase, which results in phosphorylation of the tyrosine residues of the receptor and ultimately initiates an array of signaling events [10], [11]. Besides the generation of multiple signal transduction events, the activation of EGFR by ligand also dramatically changes the cellular localization of receptors by accelerating internalization of EGFR through clathrin-dependent and -independent endocytic pathways. EGFR has been found in caveoli, Golgi, endoplasmic reticulum, lysosome-like structures, nuclear envelopes, nuclei and within mitochondria [12]–[14]. EGFR translocates to mitochondria through interaction with proteins such as cytochrome c oxidase (Cox) subunit II [12]. Demory et al. [15] hypothesized that EGF stimulation would lead to EGFR and c-Src activation followed by translocation of these molecules to the mitochondria, phosphorylation of CoxII by EGFR and/or c-Src, reduction in oxidative ATP and free radical production, and an increase in cell viability. However, mechanistic aspects of EGFR translocation to mitochondria in GBM have not been evaluated to date. EGFR has been strongly implicated in the biology of human epithelial malignancies, with therapeutic applications in cancers of the colon, head and neck, lung, and pancreas. Accordingly, the targeting of EGFR has been intensely pursued and has resulted in the development of a series of promising molecular inhibitors for use in clinical oncology and targeted therapy [16]. Suppression of EGFR expression by siRNA or inhibition of EGFR kinase activity by an agent, such as gefitinib, has already proved to be of clinical benefit in the treatment of certain cancer cell types [17]–[19]. Yao et al. [20] revealed that mitochondrial location of EGFR was independent of receptor endocytosis and that gefitinib decreased cell viability as well as the quantity of mitochondrial EGFR. Previously, we have shown that treatment of glioma cells with human umbilical cord blood stem cells (hUCBSC) inhibited the expression of XIAP, FAK and cyclin D1 with simultaneous upregulation of PTEN [21]–[24]. Based on our previous results, we hypothesized that hUCBSC could efficiently inhibit EGFR expression as well as its translocation to mitochondria. Hence, in the present study, we investigated the mitochondrial localization of EGFR expression in human GBM from several GBM patient–derived specimens and validated similar phenomenon in standard glioma cell lines. In addition, we demonstrate that EGFR translocation to mitochondria and its co-localization with FAK is highly inhibited after treatment with hUCBSC.

## Results

### EGFR co-localizes with FAK in clinical samples

Since GBM-patient derived specimens reproduce the genotypic and phenotypic characteristics of GBM more faithfully than standard glioma cell lines [25], [26], we first examined EGFR status in GBM-patient derived specimens. Using an immunohistochemistry-based strategy, we identified six GBM-patient derived specimens with high expression of EGFR as compared to normal brain specimen (Fig. 1A). The mRNA expression levels of EGFR corresponded to the immunohistochemistry results (Fig. 1B). However, compared to the expression of EGFR, we did not observe much expression of FAK in GBM-patient derived samples. On the contrary, expression of c-Src was higher in samples where EGFR expression is low (for e.g., hGBM9, hGBM13) (Fig. 1C). Next, we checked the protein levels of these molecules. EGFR protein expression levels almost correspond to the levels observed with immunohistochemistry and mRNA expression (Fig. 1D). Contrary to this, pEGFR levels can be seen in only hGBM2 and hGBM6 (Fig. 1E). On the other hand, FAK expression is seen in all the samples with faint expression in hGBM8. Higher expression of p-Fak was observed in hGBM6 and hGBM9 samples with faint expression in remaining clinical samples. c-Src expression was seen in all GBM samples with faint expression in hGBM8. Phospho-c-Src expression was observed only in hGBM2, hGBM3, hGBM9 and hGBM13 samples with very faint expression in hGBM6. Once we confirmed the presence of EGFR and FAK in GBM-patient derived samples, we checked for the co-localization of active forms of FAK and EGFR in mitochondria. In all clinical samples, co-localization of pEGFR with pFAK is clearly established in the mitochondria (Fig. 2). Having confirmed the expression of EGFR in clinical samples and its association with FAK, we evaluated the significance of hUCBSC treatment in glioma cells and xenografts in regards to EGFR status.

**Figure 1:** Expression of EGFR in GBM-patient derived specimens. (A) Control brain and GBM-patient derived specimens were subjected to DAB immunohistochemistry using anti-rabbit EGFR antibody (bar = 200 µm). (B) mRNA extracted from the above specimens was subjected to RT-PCR using primers specific for EGFR, FAK, c-Src and β-actin (loading control). (C) Quantitative analysis of (B). (D) Tissue lysates (40 µg protein) of the above specimens were subjected to Western blotting using the following antibodies: EGFR, pEGFR, FAK, pFAK, c-Src and phospho-c-Src. Mouse anti-GAPDH (1∶1000) served as the loading control. (E) Quantitative analysis of (D). *Significant at *p*<0.05 compared to control brain samples.

**Figure 2:** Colocalization of pEGFR and pFAK in clinical samples. Control brain and GBM-patient derived specimens were labeled with pEGFR and pFAK antibodies along with Mito Tracker (green) and processed for immunofluorescence. pEGFR was conjugated with Alexa Fluor 350 (blue) and pFAK was conjugated with Alexa Fluor 594 (red) secondary antibodies (bar = 100 µm).

### hUCBSC treatment inhibits EGFR

Once we confirmed the expression status of EGFR and FAK in clinical samples, we evaluated the expression levels of EGFR, FAK and other molecules in human glioma cell lines both *in vitro* and *in vivo* with reference to the treatment effect of hUCBSC in these glioma cells. Expression of EGFR is highly downregulated in hUCBSC-treated U87, U251 and 5310 glioma cells as compared to their controls (Fig. 3A). Similarly, hUCBSC significantly reduced EGFR expression in U251 and 5310 *in vivo* xenografts (Fig. 3B).

**Figure 3:** Inhibition of EGFR by hUCBSC treatment. For *in vitro* experiments, glioma cells (U251, U87 and 5310) were co-cultured with hUCBSC for 72 hours. For *in vivo* experiments, U251 (1×10^6^ cells) and 5310 (8×10^5^ cells) tumor cells were intracerebrally injected into the right side of the brain of the nude mice. Nude mice with pre-established intracranial human glioma tumors (U251 or 5310) were treated with 2×10^5^ hUCBSC by intracranial injection. Seven days after tumor implantation, the mice were injected with hUCBSC towards the left side of the brain. Fourteen days after hUCBSC administration, the brains were harvested, sectioned, and stained with appropriate antibodies. (A) U87, U251 and 5310 glioma cells alone and after co-culture with hUCBSC were labeled with mouse anti-EGFR antibody and processed for immunofluorescence. EGFR was conjugated with Alexa Fluor 488 (green) secondary antibody (n = 3; bar = 100 µm). (B) Control and hUCBSC-treated tumor sections were labeled with mouse anti-EGFR antibody and processed for DAB immunohistochemistry. For (C) and (E), total mRNA was extracted, converted to cDNA, and subjected to semi-quantitative RT-PCR. (C) Control and hUCBSC-treated U251, U87 and 5310 *in vitro* cDNAs were subjected to RT-PCR using EGFR, FAK and c-Src primers. (D) Quantitative analysis of (C). *Significant at *p*<0.05 compared to respective control glioma cells. **Significant at *p*<0.01 compared to respective control glioma cells. (E) Control and hUCBSC-treated U251 and 5310 *in vivo* cDNAs were subjected to RT-PCR using EGFR, FAK and c-Src primers. β-actin served as a loading control. (F) Quantitative analysis of (E). *Significant at *p*<0.05 compared to respective control glioma tissues. For (G) and (I), 40 µg of proteins were loaded onto 8% gels and transferred onto nitrocellulose membranes, probed with respective antibodies, and developed by autoradiography. (G) Control and hUCBSC-treated U251, U87 and 5310 glioma cell lysates were processed and immunoblotted with EGFR, FAK and c-Src antibodies. (H) Quantitative analysis of (G). **Significant at *p*<0.01, *Significant at *p*<0.05 compared to respective control glioma cells. (I) Control and hUCBSC-treated U251 and 5310 *in vivo* brain tissue lysates were processed by standard Western blotting and probed with EGFR, FAK and c-Src antibodies. GAPDH served as a loading control. (J) Quantitative analysis of (I). **Significant at *p*<0.01, *Significant at *p*<0.05 compared to respective control glioma tissue lysates. For (C–J), n≥3.

Further, we checked the expression of EGFR, FAK and c-Src in glioma cells lines and their co-cultures with hUCBSC. We observed that in co-cultures of glioma cells with hUCBSC, the mRNA levels of EGFR, FAK and c-Src are downregulated (Fig. 3C, 3D). This is associated with the downregulation of these molecules at protein levels also (Fig. 3G). We observed that EGFR and FAK are more significantly downregulated compared to c-Src (Fig. 3H). To confirm these results, we checked the expression of these molecules in nude mice brain xenografts. Similar to the *in vitro* results, in hUCBSC-treated brain tissues also, mRNAs of EGFR, FAK and c-Src were downregulated (Figs. 3E, 3F). This ultimately resulted in the lower expression of these molecules at protein levels (Figs. 3I, 3J). These results prove that hUCBSC downregulate EGFR, FAK and c-Src at both transcriptional and translational stages in both *in vitro* and *in vivo* conditions. Since EGFR plays a vital role in the proliferation of glioma cells, we tested the expression of Ki67 in U87, U251 and 5310 glioma cells. These cells express high levels of the ubiquitous proliferation marker Ki67 (Fig. 4A); treatment with hUCBSC lowered the expression of Ki67 indicating EGFR-mediated proliferation of glioma cells is inhibited by hUCBSC treatments. Further, we checked the co-localization of EGFR and FAK in glioma cells. As expected pEGFR co-localized with pFAK in glioma cells and this co-localization was completely inhibited by hUCBSC treatment (Fig. 4B). To confirm these results, we treated U251, U87 and 5310 cells with external supply of EGF and observed higher expression of EGFR and FAK as compared to control glioma cells (Fig. 4C). In another experiment, we treated glioma cells with EGF initially and then co-cultured these cells with hUCBSC for 72 hours. Even though glioma cells were supplied with exogenous EGF, hUCBSC were highly efficient in downregulating both EGFR and FAK in these treatments (Fig. 4D). To further substantiate these results, we performed cell proliferation assays based on BrdU incorporation. In all three glioma cell lines of the present study, hUCBSC inhibited cell proliferation by more than 80% (Fig. 5A). The inhibition of cell proliferation was more pronounced in hUCBSC-treated 5310 cell lines. In another experiment, we observed that exogenous supply of EGF increased cell proliferation of glioma cells by about 10% (Fig. 5B). However, hUCBSC were able to inhibit proliferation of exogenous EGF-supplied cells to <80% than control glioma cells. Further to compare and evaluate the efficiency of hUCBSC with that of Temozolomide (TMZ), we performed combination treatments of hUCBSC and TMZ on glioma cells. TMZ alone inhibited the proliferation of glioma cells to <40% (Fig. 5C). However, combination treatments of hUCBSC and TMZ at different time intervals showed profound effect on the cell proliferation of glioma cells compared to single TMZ treatments. These experiments confirm the efficacy of hUCBSC against EGF-treated glioma cells and the effect of hUCBSC in inhibiting glioma cell proliferation.

**Figure 4:** Inhibition of EGFR and FAK co-localization by hUCBSC. (A) Control and hUCBSC-treated U87, U251 and 5310 glioma cells were labeled with Ki67 antibody and processed for immunofluorescence. Ki67 was conjugated with Alexa Fluor 594 (red) secondary antibody (n≥3; bar = 100 µm). (B) Control and hUCBSC-treated U87, U251 and 5310 glioma cells were labeled with pEGFR and pFAK antibodies and processed for immunofluorescence. pFAK was conjugated with Alexa Fluor 488 (green) and pEGFR was conjugated with Alexa Fluor 594 (red) secondary antibodies (n≥3; bar = 100 µm). (C) Control, EGF-treated, EGF+hUCBSC-treated, and hUCBSC-treated U251, U87 and 5310 cells were processed and 40 µg of proteins were loaded onto 8% gels and transferred onto nitrocellulose membranes, probed with EGFR and FAK antibodies, and developed by autoradiography. GAPDH served as a loading control. n = 3. (D) Quantitative analysis of (C). *Significant at *p*<0.05 compared to respective control glioma cells by one-way ANOVA.

**Figure 5:** Inhibition of cell proliferation by hUCBSC treatments. (A) Control and hUCBSC-treated glioma cells at different time points were analyzed for cell proliferation by incorporation of BrdU. *Significant at *p*<0.05 compared to respective control cells. **Significant at *p*<0.01 compared to respective control cells (by *t*-test). (B) Control, EGF-treated and EGF+hUCBSC treated glioma cells were analyzed for cell proliferation. *Significant at *p*<0.05 both for control *vs.* EGF+hUCBSC treatment and EGF *vs.* EGF+hUCBSC treatments (one-way ANOVA followed by Bonferroni's post hoc test). (C) Control, TMZ treated, TMZ+hUCBSC treated glioma cells were subjected to cell proliferation analysis by BrdU incorporation. *Significant at *p*<0.05; **Significant at *p*<0.01 both for control *vs.* TMZ treatment and control *vs.* TMZ+hUCBSC treatments (one-way ANOVA followed by Bonferroni's post hoc test). For all these tests, raw data was taken into consideration to perform statistical analyses and then results were presented as % control values. Each bar represents n≥6.

### hUCBSC inhibits translocation of phospho-EGFR to mitochondria of glioma cells

EGFR activation stimulates many complex intracellular signaling pathways. Apart from this activation, EGFR translocates to mitochondria and co-localizes with FAK to further activate mitochondria-mediated signaling in glioma cells. Since we observed that hUCBSC treatments inhibited EGFR expression in glioma cells, we decided to further evaluate translocation of the active form of EGFR to mitochondria in glioma cells. In all these cell lines, translocation of activated EGFR to mitochondria was inhibited by hUCBSC treatments (Fig. 6A). Similarly, *in vivo* samples also show inhibition of translocation of pEGFR to mitochondria (Fig. 6B). Thus, under both *in vitro* and *in vivo* conditions, hUCBSC prevented the translocation of pEGFR to mitochondria. As mentioned earlier, activation of EGFR stimulates activation of many different proteins like FAK and c-Src. We therefore evaluated the expression of phospho-c-Src in mitochondria of glioma cells. All of the glioma cell lines in the present study showed higher expression of phospho-c-Src (Fig. 6C). We also observed higher expression of phospho-c-Src *in vivo* in nude mice brain tumors (Fig. 6D). In both cases, the expression of phospho-c-Src was inhibited by hUCBSC treatments. To confirm these results, we ran Western immunoblots of pEGFR, pFAK and p-c-Src in whole cell lysates and whole tissue lysates of control and hUCBSC-treated glioma samples. We observed downregulation of phosphorylated forms of EGFR, FAK and c-Src in hUCBSC-treated glioma cells (Fig. 7A). Downregulation of active forms of EGFR and c-Src are more significant compared to FAK in these cell lysates (Fig. 7B). In a similar fashion, these active forms were also downregulated in hUCBSC-treated total tissue lysates of brain xenografts (Figs. 7C, 7D). Compared to total tissue lysates, the mitochondrial fractions of brain xenografts showed high concentration of phospho-forms of EGFR, FAK and c-Src (Figs. 7E, 7F). The mitochondrial fractions of U251 control tissues show 68.49±0.42% (mean ± S.D.) of pEGFR whereas 5310 control tissues show about 53.72±2.21% of pEGFR, which means that out of total pEGFR present in these glioma tissues, major portion of activated EGFR is translocated to mitochondria (Fig. 7E). The mitochondrial fractions of hUCBSC treated U251 tissues show 33.21±1.52% of pEGFR whereas hUCBSC treated 5310 tissues show about 24.39±0.53% of pEGFR, which means that hUCBSC inhibited the translocation of pEGFR to mitochondria. Since, endosomal-lysosomal internalization upon translocation of activated plasma membrane bound EGFR takes place, we tested this pathway by immunohistochemistry methods. Probing the control and hUCBSC-treated nude mice brain sections with Cathepsin-L antibody, we observed that Cathepsin-L is highly activated in U251 and 5310 xenograft tumors, and the expression is highly downregulated in hUCBSC treatments (Fig. S1). These results confirm that hUCBSC are efficient in inhibiting the phosphorylation of EGFR, FAK and c-Src in glioma cells and tissues, thereby preventing the translocation of EGFR to mitochondria as well as interaction of EGFR with FAK and c-Src.

**Figure 6:** Downregulation of pEGFR and phospho-c-Src in mitochondria in hUCBSC treatments. (A) Control and hUCBSC-treated U251, U87 and 5310 cells were labeled with pEGFR and Mito Tracker green and processed for immunofluorescence. (B) Control and hUCBSC-treated U251 and 5310 tissue sections were labeled with pEGFR and Mito Tracker green and processed for immunofluorescence. pEGFR was conjugated with Alexa Fluor 594 (red) secondary antibody (n≥3; bar = 100 µm). (C) Control and hUCBSC-treated U251, U87 and 5310 cells were labeled with phospho-c-Src and Mito Tracker green and processed for immunofluorescence. (D) Control and hUCBSC-treated U251 and 5310 tissue sections were labeled with phospho-c-Src and Mito Tracker green and processed for immunofluorescence. Phospho-c-Src was conjugated with Alexa Fluor 594 (red) secondary antibody (n≥3; bar = 100 µm).

**Figure 7:** Downregulation of EGFR-mediated signaling molecules in hUCBSC treatments. For (A), (C), (E), (G) and (I) 40 µg of proteins were loaded onto 8–12% gels and transferred onto nitrocellulose membranes, probed with respective antibodies, and developed by autoradiography. (A) *In vitro* samples probed with pEGFR, pFAK, p-c-Src and GAPDH. (B) Quantitative analysis of (A). *Significant at *p*<0.05 compared to respective control glioma cells. (C) *In vivo* cytosolic fractions probed with pEGFR, pFAK, p-c-Src and GAPDH. n = 3. (D) Quantitative analysis of (C). *Significant at *p*<0.05 compared to respective control glioma tissues. (E) *In vivo* mitochondrial fractions probed with pEGFR, pFAK, p-c-Src and Cox IV. n = 3. (F) Quantitative analysis of (E). *Significant at *p*<0.05 compared to respective control glioma tissues. Control and hUCBSC-treated U251, U87 and 5310 glioma cell lysates (G) and control and hUCBSC-treated U251 and 5310 glioma tissue lysates (I) were processed for immunoblotting and probed with MEK1, RAF1, Stat3 and PI3K antibodies. GAPDH served as a loading control. (H) Quantitative estimation of (G). *Significant at *p*<0.05 compared to respective glioma control cells. **Significant at *p*<0.01 compared to respective glioma control cells. (J) Quantitative estimation of (I). *Significant at *p*<0.05 compared to respective glioma control tissues. **Significant at *p*<0.01 compared to respective glioma control tissues. (K) Tumor size volume estimated in control and hUCBSC treated nude mice brains. *Significant at *p*<0.05 compared to glioma controls. Error bars indicate ± SD. For (A) to (K), n≥3.

Finally, we assessed the expression of EGFR signaling molecules in glioma cells *in vitro* and *in vivo* tumors after treatment with hUCBSC. The main pathways stimulated by the EGFR are the mitogen-activated protein kinases (MAPK), the phosphatidylinositol 3-kinase–AKT, and signal transducer and activator of transcription proteins (STAT), such as STAT3 [27]. In addition, the activation of STAT3 also relies on the recruitment of the Src kinase to the EGFR [28], [29]. Upon nuclear translocation, the STAT3 transcription factor up-regulates several genes involved in cell cycle progression [30], [31], cell survival [32] and metastasis [33]. Another molecule of EGFR signaling cascade RAF1 protein, can phosphorylate to activate the dual specificity protein kinases MEK1 and MEK2, which in turn phosphorylate to activate the serine/threonine specific protein kinases, ERK1 and ERK2. These key molecules of EGFR signaling MEK1, RAF1, STAT3 and PI3K were downregulated in hUCBSC treated glioma cells (Fig. 7G). Quantitative analysis shows that both RAF1 and PI3k (p<0.01) show significant downregulation compared to MEK1 and STAT3 (p<0.05) (Fig. 7H). We also checked the expression of these molecules in hUCBSC-treated glioma tumors *in vivo* and observed that these EGFR signaling molecules are downregulated compared to untreated tumors (Fig. 7I). Similar to our *in vitro* results, RAF1 and PI3k (p<0.01) molecules show significant downregulation compared to MEK1 and STAT3 (p<0.05) by hUCBSC treatments (Fig. 7J). Finally, we observed tumor size regression by about 75% in hUCBSC-treated *in vivo* nude mice brains of both U251 and 5310 xenografts (Fig. 7K). Our results show that hUCBSC has the ability to downregulate the expression of multiple members of EGFR signaling cascades, in both *in vitro* and *in vivo* conditions.

## Discussion

Overexpression of EGFR is one of the most frequently diagnosed genetic aberrations of glioblastoma multiforme (GBM). EGFR signaling is involved in diverse cellular functions and is dependent on the type of preferred receptor complexes. EGFR activation stimulates many complex intracellular signaling pathways that are tightly regulated by the presence and identity of the ligand, heterodimer composition, and the availability of phosphotyrosine-binding proteins. The two primary signaling pathways activated by EGFR include the RAS/RAF/MEK/ERK and the PI3K/AKT axes; however, Src tyrosine kinases, PlCγ, PKC, and STAT activation and downstream signaling have also been well documented [16], [34], [35]. EGFR gene amplification is one of the most common genetic changes in GBM and can lead to the activation of various downstream signaling molecules, including STAT3, MAPK, and AKT [36]. Receptor phosphorylation leads to the recruitment of multiple effector proteins through recognition and binding of Src homology 2 (SH2) and phosphotyrosine binding (PTB) domains on the effector proteins to phosphotyrosine motifs on the receptor [37]. The formation of this signaling complex results in the initiation of various downstream signaling cascades, including the phosphoinositide-3-kinase (PI3K), mitogen-activated protein kinase (MAPK), and signal transducer and activator of transcription 3 (STAT3) pathways, which regulate a multitude of cellular responses. To evaluate the signaling pathways mediated by EGFR, we determined the expression of EGFR in GBM-patient derived specimens. Our results confirm that immunohistochemically detectable EGFR is overexpressed in some grade IV glioblastoma samples. These results are in correlation with transcriptional and translational status of EGFR expression. However, in regards to the clinical outcome, EGFR expression did not correlate with other molecules like FAK. EGFR staining was negative in the normal brain samples and these results suggest that EGFR expression is an indicator of a malignant phenotype of the majority of GBM. Co-overexpression of EGFR, FAK and c-Src frequently occurs in human tumors and is linked to enhanced tumor growth [38], [39]. In the present study, we also observed co-localization of EGFR with FAK in mitochondria of GBM-patient derived specimens, which is indicative of the roles of EGFR, FAK and mitochondria in enhanced tumor growth.

In recent years, EGFR has become a promising target for therapies for different tumors. The poor prognosis of GBM patients is due in part to classical chemo- and radioresistance properties demonstrated by these tumors. Newly diagnosed GBM patients typically undergo surgical resection of the tumor followed by concomitant temozolamide (TMZ) treatment and radiotherapy and subsequent administration of TMZ for 6 months as adjuvant chemotherapy [40]. Because EGFRvIII has been shown to contribute to tumor progression and chemo-radioresistance, an attractive strategy would be to develop targeted therapeutics against this receptor for use as a monotherapy, thereby minimizing the systemic side effects of whole-brain irradiation and TMZ administration, especially because genetic manipulation of EGFRvIII has resulted in tumor shrinkage in a preclinical setting [8]. The monoclonal anti-EGFR antibody cetuximab and the EGFR tyrosine kinase inhibitor erlotinib led (in monotherapy or in combination with cytotoxic drugs) to improved survival in patients with colorectal cancer, non-small cell lung cancer and advanced pancreatic cancer [41]–[43]. Based on these earlier reports and our successful results with GBM tumor regression by hUCBSC, we hypothesized that hUCBSC could efficiently downregulate the expression of EGFR and its signaling molecules. Previously, we reported that hUCBSC inhibit FAK expression and its related angiogenesis in GBM *in vitro* and *in vivo* [22]. In the present study, we observed downregulation of EGFR expression in glioma cells. Even when we supplied exogenous EGF, which increases EGFR expression of glioma cells in a drastic manner, treatment with hUCBSC efficiently inhibited the expression of both EGFR and FAK in these cells.

Although generally represented as a plasma membrane protein, EGFR has been found in the nucleus and sub-cellular organelles. Recently, the mitochondrial localization of the EGFR was reported. Mitochondria are involved in diverse cellular and metabolic processes including proliferation, programmed cell death execution and signal transduction [44]–[46]. Recent reports reveal that there exists an integrated signal system in the mitochondrion to coordinate the various molecular messages that enter and exit the mitochondrion according to the diverse needs of the cell [47]–[49]. Protein kinases, protein phosphatases, and even transcriptional factors, which are not conventionally mitochondrial resident members, are revealed to have a mitochondrial location [44], [48]. However, the molecular mechanisms underlying EGFR localization in mitochondria remain largely unknown. EGFR mitochondrial localization is regulated by either autophagy or programmed cell death and is correlated with cell survival [50]. Demory et al. [15] postulated that EGF stimulation would lead to EGFR and c-Src activation followed by translocation of these molecules to the mitochondria, phosphorylation of CoxII by EGFR and/or c-Src, reduction in oxidative ATP and free radical production, and an increase in cell viability. Mitochondrial-localized EGFR is independent of its internalization and may be correlated with cell survival and participate in the ligand-induced programmed cell death [20]. In our studies, we observed that phosphorylation of EGFR is inhibited by hUCBSC treatments. Unless EGFR is activated, it cannot translocate to mitochondria or any other sub-cellular organelles. Hence, we could not observe translocation of EGFR to mitochondria in hUCBSC-treated *in vitro* and *in vivo* samples. Further, we did not observe any co-localization of activated EGFR and FAK molecules in mitochondria after hUCBSC treatments.

In summary, our data indicate that hUCBSC coordinately regulates EGFR signaling at cytosolic and mitochondrial levels in glioma cells. The effect of hUCBSC action is to inhibit cell cycle progression and reduce cell growth and viability as reported previously. The reported down-regulation of EGFR in GBM tumors, together with the ability to regulate oncogenic EGFR signaling in glioma cell lines, suggests the therapeutic potential of hUCBSC in regulating GBM tumors. The inhibition of EGFR by hUCBSC can be effective in the treatment of GBM. Our previous findings indicated that hUCBSC can inhibit cell viability by initially reducing the content of mitochondrial membrane potential [21]. The results of the present study show that inhibition of EGFR localization to mitochondria provide further evidence of the growth inhibitory effect of hUCBSC on glioma cells. Our findings show that hUCBSC inhibit EGFR localization in mitochondria in GBM cells and provide relevant preclinical information that can be exploited for the development of effective hUCBSC-based therapies.

## Materials and Methods

### Ethics Statement

After obtaining informed consent, human umbilical cord blood was collected from healthy volunteers according to a protocol approved by the Peoria Institutional Review Board, Peoria, IL, USA. The consent was written and approved. The approved protocol number is 06-014, dated December 10, 2009 and renewed on November 11, 2010. The Institutional Animal Care and Use Committee of the University Of Illinois College Of Medicine at Peoria, Peoria, IL, USA approved all surgical interventions and post-operative animal care. The consent was written and approved. The approved protocol number is 851, dated November 20, 2009 and renewed on March 15, 2011.

### Cell cultures

Two high-grade human glioma cell lines (U251, U87) and one xenograft cell line (5310) were used for this study. U251 and U87 cells were obtained from American Type Culture Collection (ATCC, Manassas, VA). The 5310 xenograft cell line was kindly provided by Dr. David James at University of California, San Francisco. U251 and U87 cells were grown in DMEM supplemented with 10% fetal bovine serum (FBS) (Hyclone, Logan, UT) and 1% penicillin-streptomycin (Invitrogen, Carlsbad, CA). The 5310 xenograft cell line was grown in RPMI 1640 medium supplemented with 10% FBS and 1% penicillin-streptomycin. For hUCBSC, after obtaining informed consent, human umbilical cord blood was collected from healthy volunteers according to a protocol approved by the University Of Illinois College Of Medicine at Peoria Institutional Review Board. Cord blood was processed as described previously by sequential Ficoll density gradient purification [51]. Next, we selected cells using CD29^+^ and CD81^+^ markers as described previously. The nucleated cells were grown in mesencult medium (Stem Cell Technologies, Vancouver, Canada) supplemented with 20% FBS and 1% penicillin-streptomycin and plated in 100-mm culture dishes. All the cells were grown at 37°C in an incubator with a 5% CO_2_ atmosphere. For co-culture experiments, hUCBSC and glioma cells were cultured at a ratio of 1∶1 (1×10^6^ for each cell line) for 72 hours. Co-cultures of hUCBSC and U251, hUCBSC and U87 were grown in DMEM (with 10% FBS) and co-cultures of hUCBSC and 5310 were grown in RPMI-1640 (with 10% FBS) and then FACS sorted as described previously [24].

### Collection of patients' specimens

GBM specimens were collected from patients with histologic diagnosis of primary GBM (WHO grade IV astrocytoma) in accordance with the protocol approved by the University Of Illinois College Of Medicine at Peoria Institutional Review Board. Tumor diagnosis and grading were blind-reviewed by a neuropathologist. Samples that did not satisfy the inclusion criteria of primary GBM (e.g., GBM with oligodendroglioma features) were excluded from the study.

### BrdU assay for cell proliferation

Cell proliferation analysis was performed using Cell Proliferation ELISA (colorimetric) BrdU incorporation assay (Roche diagnostics, Indianapolis, IN) according to the manufacturer's protocol. Cells (0.5×10^4^ cells/well) were cultured in 96-well plates for different time periods (48 h, 72 h and 96 h for coculture treatments with hUCBSC) and treatments and incubated for 12 hours with BrdU reagent. An anti-BrdU antibody was added, and the immune complexes were detected by subsequent substrate reaction. The reaction product was quantified as per manufacturer's instructions.

### EGF and TMZ treatments

Glioma cells were subjected to serum starvation for 3 hours and then treated with EGF (100 ng/mL) for 1 hour in serum free medium. After EGF treatment, the cells were washed twice with PBS and harvested. In another experiment, glioma cells that were given EGF treatment were co-cultured with hUCBSC in 1∶1 ratio for 72 hours as described above. For Temozolomide (TMZ) treatments, the glioma cells were subjected to serum starvation for 3 hours and then treated with TMZ (1000 µM) for 24 h in serum free medium. In combination treatments with hUCBSC, stem cell treatments were given at different time periods (48 h, 72 h and 96 h) either before or after treatment with TMZ. In both EGF and TMZ treatments, we tested different concentrations and time periods and finally selected the above time points and concentrations which yield optimum results (data not shown).

### RNA analysis

Total RNA from GBM patient-derived tumor specimens (frozen) and from control and hUCBSC-treated glioma cell lines was extracted using the RNeasy Mini Kits (Qiagen, Valencia, CA). cDNA was obtained by using Transcriptor first-strand cDNA synthesis kit (Roche, Indianapolis, IN) by reverse transcription-based PCR (RT-PCR). All cDNAs were normalized to the β-actin RT-PCR product. PCR amplification was performed using the primer sets listed below, amplified by 35 cycles of PCR (94°C, 1 min; 60°C, 1 min; 72°C, 1 min) using 20 pM of specific primers.

### Primers used for RT-PCR

EGFR Forward 5′ccaagggagtttgtggagaa3′

    Reverse 5′cttccagaccagggtgttgt3′

FAK Forward 5′ggtgcaatggagcgagtatt3′

  Reverse 5′gccagtgaacctcctctga3′

c-Src Forward 5′gggtagcaacaagagcaa3′

  Reverse 5′gagttgaagcctccgaacag3′

β-Actin Forward 5′ggcatcctcaccctgaagta3′

  Reverse 5′ggggtgttgaaggtctcaaa3′

### Immunoblot analysis

Single and co-cultures of glioma cells or nude mice brain tissues (frozen) were harvested and homogenized in four volumes of homogenization buffer as described previously [51]. Samples (40–50 µg of total protein/well) were subjected to 8–12% SDS-PAGE and transferred onto nitrocellulose membranes. The reaction was detected using Hyperfilm-MP autoradiography film (Amersham, Piscataway, NJ). The following antibodies were used for Western blot analysis: mouse anti-EGFR (1∶500), goat anti-pEGFR (1∶500), mouse anti-FAK (1∶500), goat anti-phospho-FAK (1∶500), mouse anti-c-Src (1∶500), mouse anti-MEK1 (1∶500), rabbit anti-RAF1 (1∶500), mouse anti-STAT3 (1∶500), mouse anti-PI3K (1∶500) (all from Santa Cruz Biotechnology, Santa Cruz, CA), and rabbit anti-phospho-c-Src (1∶1000; Cell Signaling). Immunoreactive bands were visualized using chemiluminescence ECL Western blotting detection reagents (Amersham). Immunoblots were stripped and redeveloped with GAPDH antibody [mouse anti-GAPDH (1∶1000; Santa Cruz)] to ensure equal loading levels. Experiments were performed in triplicate. The bands in each blot were quantified using ImageJ software and the values were expressed in relation of GAPDH values.

### Intracranial tumor growth inhibition

The Institutional Animal Care and Use Committee of the University Of Illinois College Of Medicine at Peoria approved all surgical interventions and post-operative animal care. For the intracerebral tumor model, U251 (1×10^6^ cells) and 5310 (8×10^5^ cells) tumor cells were intracerebrally injected into the right side of the brain of the nude mice as described previously [23]. Seven days after tumor implantation, the mice were injected with hUCBSC in the contralateral left brain hemisphere. The ratio of the hUCBSC to cancer cells was maintained at 1∶4. Three weeks after tumor inoculation, six mice from each group were sacrificed by cardiac perfusion with 4% formaldehyde in PBS, their brains were removed, and paraffin sections were prepared. Sections were stained with H&E to visualize tumor cells and to examine tumor volume. The sections were blindly reviewed and scored semiquantitatively for tumor size. Whole-mount images of brains were also taken to determine infiltrative tumor morphology. The average tumor area per section integrated to the number of sections where the tumor was visible was used to calculate tumor volume and compared between controls and treated groups. Immunoblot analyses and RT-PCR were carried out on fresh brain tissues.

### Immunostaining analyses

GBM patient-derived specimens and brains of control and hUCBSC-treated mice were fixed in formaldehyde and embedded in paraffin as per standard protocols. Sections were deparaffinized and blocked in 1% BSA in PBS for 1 hour, and the sections were subsequently transferred to primary antibody diluted in either 1% BSA (for pEGFR and pFAK antibodies) or 10% normal goat serum (1∶100) (for all other antibodies). Sections were allowed to incubate in the primary antibody solution overnight at 4°C in a humidified chamber. Sections were then washed in PBS and placed in either 1% BSA or 10% goat serum with the appropriate secondary antibody. The sections were incubated with the secondary antibody for 1 hour and visualized using a confocal microscope. Transmitted light images were obtained after H&E staining as per standard protocol to visualize the morphology of the sections. Negative controls were maintained without primary antibody or by using IgG fraction. For DAB immunohistochemistry, sections were probed with antibodies and then stained with DAB (Sigma) and further stained with Hematoxylin. For immunofluorescence studies, cultured glioma cells plated in 2-well chamber slides were rinsed twice with phosphate buffered saline (PBS) and fixed in 4% paraformaldehyde. After additional PBS rinses, cells were blocked with 1× PBS with 1% bovine serum albumin (BSA) for 1 hour. Primary antibodies (1∶100 dilutions) were diluted in either 10% goat serum or 1% BSA and applied overnight at 4°C. Alexa Fluor-conjugated secondary antibodies were diluted (1∶200) in either 10% goat serum or 1% BSA and applied individually for 1 hour at room temperature. We used the following antibodies: mouse anti-EGFR, mouse anti-Ki67, rabbit anti-FAK, goat anti-pEGFR, mouse anti-phospho-c-Src (all from Santa Cruz Biotechnology). For mitochondrial localization, we used Mito Tracker Green (Invitrogen) as per the manufacturer's instructions. Before mounting, the cells were stained with 4′, 6-diamidino-2-phenylindole (DAPI). The cells were observed using a fluorescence microscope (Olympus IX71, Olympus, Melville, NY) and/or a confocal microscope (Olympus Fluoview) and photographed. We used same antibodies for both immunofluorescence studies and immunohistochemistry studies. Negative controls were maintained without primary antibody or by using IgG fraction.

### Statistical analyses

Values are shown as mean ± SD of at least three independent experiments. Results were analyzed using a two-tailed Student's *t*-test using Graph Pad Prism version 3.02, a statistical software package. Results were considered statistically significant at *p*<0.05 or *p*<0.01. For comparing more than two groups, statistical significance using one way analysis of variance (ANOVA) was used. Data for each treatment group were represented as mean ± SEM and compared with other groups for significance by one-way ANOVA followed by Bonferroni's post hoc test (multiple comparison tests) using Graph Pad Prism version 3.02. Results were considered statistically significant at a *p*<0.05 or *p*<0.01.

## Supporting Information

Figure S1 **Inhibition of lysosomal internalization by hUCBSC treatments.** Control and hUCBSC-treated nude mice brain sections were immunoprobed with mouse anti-Cathepsin L antibody and processed for DAB staining followed by Hematoxylin staining. Bar = 200 µm. n≥3.
(TIF)

## References

[1] Furnari FB, Fenton T, Bachoo RM, Mukasa A, Stommel JM (2007). Malignant astrocytic glioma: genetics, biology, and paths to treatment.. Genes Dev.

[2] Heimberger AB, Suki D, Yang D, Shi W, Aldape K (2005). The natural history of EGFR and EGFRvIII in glioblastoma patients.. J Transl Med.

[3] Layfield LJ, Willmore C, Tripp S, Jones C, Jensen RL (2006). Epidermal growth factor receptor gene amplification and protein expression in glioblastoma multiforme: prognostic significance and relationship to other prognostic factors.. Appl Immunohistochem Mol Morphol.

[4] Ohgaki H, Kleihues P (2005). Population-based studies on incidence, survival rates, and genetic alterations in astrocytic and oligodendroglial gliomas.. J Neuropathol Exp Neurol.

[5] Frederick L, Wang XY, Eley G, James CD (2000). Diversity and frequency of epidermal growth factor receptor mutations in human glioblastomas.. Cancer Res.

[6] Cancer Genome Atlas Research Network collaborators (2008). Comprehensive genomic characterization defines human glioblastoma genes and core pathways.. Nature.

[7] Parsons DW, Jones S, Zhang X, Lin JC, Leary RJ (2008). An integrated genomic analysis of human glioblastoma multiforme.. Science.

[8] Huang PH, Xu AM, White FM (2009). Oncogenic EGFR signaling networks in glioma.. Sci Signal.

[9] Hatanpaa KJ, Burma S, Zhao D, Habib AA (2010). Epidermal growth factor receptor in glioma: signal transduction, neuropathology, imaging, and radioresistance.. Neoplasia.

[10] Schlessinger J (2000). Cell signaling by receptor tyrosine kinases.. Cell.

[11] Waterman H, Yarden Y (2001). Molecular mechanisms underlying endocytosis and sorting of ErbB receptor tyrosine kinases.. FEBS Lett.

[12] Boerner JL, Demory ML, Silva C, Parsons SJ (2004). Phosphorylation of Y845 on the epidermal growth factor receptor mediates binding to the mitochondrial protein cytochrome c oxidase subunit II.. Mol Cell Biol.

[13] Carpentier JL, Rees AR, Gregoriou M, Kris R, Schlessinger J (1986). Subcellular distribution of the external and internal domains of the EGF receptor in A-431 cells.. Exp Cell Res.

[14] Lin SY, Makino K, Xia W, Matin A, Wen Y (2001). Nuclear localization of EGF receptor and its potential new role as a transcription factor.. Nat Cell Biol.

[15] Demory ML, Boerner JL, Davidson R, Faust W, Miyake T (2009). Epidermal growth factor receptor translocation to the mitochondria: regulation and effect.. J Biol Chem.

[16] Wheeler DL, Dunn EF, Harari PM (2010). Understanding resistance to EGFR inhibitors-impact on future treatment strategies.. Nat Rev Clin Oncol.

[17] Fan QW, Weiss WA (2005). RNA interference against a glioma-derived allele of EGFR induces blockade at G2M.. Oncogene.

[18] Friedmann BJ, Caplin M, Savic B, Shah T, Lord CJ (2006). Interaction of the epidermal growth factor receptor and the DNA-dependent protein kinase pathway following gefitinib treatment.. Mol Cancer Ther.

[19] Smith K, Gunaratnam L, Morley M, Franovic A, Mekhail K (2005). Silencing of epidermal growth factor receptor suppresses hypoxia-inducible factor-2-driven VHL−/− renal cancer.. Cancer Res.

[20] Yao Y, Wang G, Li Z, Yan B, Guo Y (2010). Mitochondrially localized EGFR is independent of its endocytosis and associates with cell viability.. Acta Biochim Biophys Sin (Shanghai).

[21] Dasari VR, Velpula KK, Kaur K, Fassett D, Klopfenstein JD (2010). Cord Blood Stem Cell-Mediated Induction of Apoptosis in Glioma Downregulates X-Linked Inhibitor of Apoptosis Protein (XIAP).. PLoS One.

[22] Dasari VR, Kaur K, Velpula KK, Dinh DH, Tsung AJ (2010). Downregulation of Focal Adhesion Kinase (FAK) by cord blood stem cells inhibits angiogenesis in glioblastoma.. Aging (Albany NY).

[23] Dasari VR, Kaur K, Velpula KK, Gujrati M, Fassett D (2010). Upregulation of PTEN in glioma cells by cord blood mesenchymal stem cells inhibits migration via downregulation of the PI3K/Akt pathway.. PLoS One.

[24] Velpula KK, Dasari VR, Tsung AJ, Gondi CS, Klopfenstein JD (2011). Regulation of glioblastoma progression by cord blood stem cells is mediated by downregulation of cyclin D1.. PlosOne.

[25] Galli R, Binda E, Orfanelli U, Cipelletti B, Gritti A (2004). Isolation and characterization of tumorigenic, stem-like neural precursors from human glioblastoma.. Cancer Res.

[26] Lee J, Kotliarova S, Kotliarov Y, Li A, Su Q (2006). Tumor stem cells derived from glioblastomas cultured in bFGF and EGF more closely mirror the phenotype and genotype of primary tumors than do serum-cultured cell lines.. Cancer Cell.

[27] Grandis JR, Drenning SD, Chakraborty A, Zhou MY, Zeng Q (1998). Requirement of Stat3 but not Stat1 activation for epidermal growth factor receptor- mediated cell growth In vitro.. J Clin Invest.

[28] Olayioye MA, Beuvink I, Horsch K, Daly JM, Hynes NE (1999). ErbB receptor-induced activation of stat transcription factors is mediated by Src tyrosine kinases.. J Biol Chem.

[29] Biscardi JS, Maa MC, Tice DA, Cox ME, Leu TH (1999). c-Src-mediated phosphorylation of the epidermal growth factor receptor on Tyr845 and Tyr1101 is associated with modulation of receptor function.. J Biol Chem.

[30] Barre' B, Vigneron A, Coqueret O (2005). The STAT3 transcription factor is a target for the Myc and riboblastoma proteins on the Cdc25A promoter.. J Biol Chem.

[31] Leslie K, Lang C, Devgan G, Azare J, Berishaj M (2006). Cyclin D1 is transcriptionally regulated by and required for transformation by activated signal transducer and activator of transcription 3.. Cancer Res.

[32] Ivanov VN, Bhoumik A, Krasilnikov M, Raz R, Owen-Schaub LB (2001). Cooperation between STAT3 and c-jun suppresses Fas transcription.. Mol Cell.

[33] Dechow TN, Pedranzini L, Leitch A, Leslie K, Gerald WL (2004). Requirement of matrix metalloproteinase-9 for the transformation of human mammary epithelial cells by Stat3-C.. Proc Natl Acad Sci USA.

[34] Marmor MD, Skaria KB, Yarden Y (2004). Signal transduction and oncogenesis by ErbB/HER receptors.. Int J Radiat Oncol Biol Phys.

[35] Yarden Y, Sliwkowski MX (2001). Untangling the ErbB signaling network.. Nat Rev Mol Cell Biol.

[36] Mizoguchi M, Betensky RA, Batchelor TT, Bernay DC, Louis DN (2006). Activation of STAT3, MAPK, and AKT in malignant astrocytic gliomas: correlation with EGFR status, tumor grade, and survival.. J Neuropathol Exp Neurol.

[37] Jones RB, Gordus A, Krall JA, MacBeath G (2006). A quantitative protein interaction network for the ErbB receptors using protein microarrays.. Nature.

[38] Biscardi JS, Ishizawar RC, Silva CM, Parsons SJ (2000). Tyrosine kinase signaling in breast cancer: epidermal growth factor receptor and c-Src interactions in breast cancer.. Breast Cancer Res.

[39] Ishizawar R, Parsons SJ (2004). c-Src and cooperating partners in human cancer.. Cancer Cell.

[40] Stupp R, Dietrich PY, Ostermann Kraljevic S, Pica A, Maillard I (2002). Promising survival for patients with newly diagnosed glioblastoma multiforme treated with concomitant radiation plus temozolomide followed by adjuvant temozolomide.. J Clin Oncol.

[41] Cunningham D, Humblet Y, Siena S, Khayat D, Bleiberg H (2004). Cetuximab monotherapy and cetuximab plus irinotecan in irinotecan-refractory metastatic colorectal cancer.. N Engl J Med.

[42] Moore MJ, Goldstein D, Hamm J, Figer A, Hecht JR (2007). Erlotinib plus gemcitabine compared with gemcitabine alone in patients with advanced pancreatic cancer: a phase III trial of the National Cancer Institute of Canada Clinical Trials Group.. J Clin Oncol.

[43] Shepherd FA, Rodrigues PJ, Ciuleanu T, Tan EH, Hirsh V (2005). Erlotinib in previously treated non-small-cell lung cancer.. N Engl J Med.

[44] Bonawitz ND, Clayton DA, Shadel GS (2006). Initiation and beyond: multiple functions of the human mitochondrial transcription machinery.. Mol Cell.

[45] Goldenthal MJ, Marin-Garcia J (2004). Mitochondrial signaling pathways: a receiver/integrator organelle.. Mol Cell Biochem.

[46] Newmeyer DD, Ferguson-Miller S (2003). Mitochondria: releasing power for life and unleashing the machineries of death.. Cell.

[47] Hajnoczky G, Hoek JB (2007). Cell signaling. Mitochondrial longevity pathways.. Science.

[48] Salvi M, Brunati AM, Toninello A (2005). Tyrosine phosphorylation in mitochondria: a new frontier in mitochondrial signaling.. Free Radic Biol Med.

[49] Satrustegui J, Pardo B, Del AA (2007). Mitochondrial transporters as novel targets for intracellular calcium signaling.. Physiol Rev.

[50] Yue X, Song W, Zhang W, Chen L, Xi Z (2008). Mitochondrially localized EGFR is subjected to autophagic regulation and implicated in cell survival.. Autophagy.

[51] Dasari VR, Veeravalli KK, Saving KL, Gujrati M, Klopfenstein JD (2008). Neuroprotection by cord blood stem cells against glutamate-induced apoptosis is mediated by Akt pathway.. Neurobiol Dis.

